# Role and Mechanism of circ_0058063/miR-635 Axis in the Malignant Phenotype of Multiple Myeloma RPMI8226 Cells

**DOI:** 10.1155/2021/4630934

**Published:** 2021-09-13

**Authors:** Xiaoya Li, Lingzhi Ding, Geyu Gu, Changjun Zheng, Chenshuai Pan, Qi Zheng, Ting Xiang

**Affiliations:** ^1^Department of Orthopedic, Taizhou Central Hospital (Taizhou University Hospital), Taizhou, Zhejiang 318000, China; ^2^Department of Nutrition, Taizhou First people's Hospital, Taizhou, Zhejiang 318020, China

## Abstract

**Objective:**

This study aims to explore circ_0058063 effect on multiple myeloma cells malignant phenotype and its feasible mechanism.

**Methods:**

We selected 47 cases of multiple myeloma tissues and 47 cases of normal bone marrow tissues and then used RT-qPCR method to test circ_0058063 and miR-635 expression in the tissues. Myeloma cells RPMI8226 were transfected with si-circ_0058063, miR-635 mimic, and si-circ_0058063 + anti-miR-635, respectively. Then, we adopt CCK-8 method, flow cytometry method, and Transwell and western blot methods to detect the influences of knockdown of circ_0058063 or miR-635 overexpression on RPMI8226 cell proliferation, apoptosis, migration, and invasion and also Ki-67, Bax, Bcl-2, MMP-2, and MMP-9 protein expression. The dual luciferase reporter gene assay experiment proved that it has regulatory relationship between circ_0058063 and miR-635.

**Results:**

circ_0058063 expression of multiple myeloma was higher than that in normal bone marrow tissue (*P* < 0.05), while miR-635 expression was lower than that in normal bone marrow tissue (*P* < 0.05). Knockdown of circ_0058063 or overexpression of miR-635 could reduce proliferation capacity, migration, invasion cell quantities, and Ki-67, MMP-2, MMP-9, and Bcl-2 protein expression (*P* < 0.05), while increasing apoptosis rate together with Bax protein expression (*P* < 0.05). circ_0058063 targets to negatively regulate miR-635, while knocking down miR-635 reverses the influences of knocking down circ_0058063 on RPMI8226 proliferation, apoptosis, migration, and invasion.

**Conclusion:**

circ_0058063 expression increased in multiple myeloma tissues. Knocking down its expression may inhibit myeloma proliferation, migration, and invasion by targeting and upregulating miR-635 and also promote cell apoptosis. As for multiple myeloma treatment, circ_0058063/miR-635 may provide new molecular targets.

## 1. Introduction

Multiple myeloma is known as a kind of malignant plasma cell disease. In recent years, its incidence has been increasing year by year, and it is showing a younger trend [1]. At present, the pathogenesis of multiple myeloma is not fully understood, and effective treatment methods are lacking. Therefore, exploring the abnormally expressed gene molecules in multiple myeloma and their influence on the occurrence and development of multiple myeloma can provide molecular targets for its targeted therapy. Circular RNA (circRNA) and microRNA (miRNA) are two types of noncoding RNAs. As competitive endogenous RNA, circRNA together with miRNA regulate miRNA target genes expression and then affect cell proliferation, apoptosis, and migration, which has close relationship with the occurrence and development of tumor [2, 3]. Research has shown that circ_0058063 expression is upregulated in esophageal squamous cell carcinoma, knocking down its expression can reduce the esophageal squamous cell carcinoma proliferation rate through inhibiting GLUT1 expression [4]; circ_0058063 is overexpressed in bladder cancer tissues. Knockout of circ_0058063 can markedly reduce bladder cancer cells proliferation and invasiveness, promote cell apoptosis, which may target together with miR-486-3p and inhibit FOXP4 expression, and provide a new target for bladder cancer targeted therapy [5]. However, the influences of circ_0058063 on malignant phenotype of multiple myeloma cells and its mechanism are still unknown. Circular RNA Interactome bioinformatics software predicts that circ_0058063 may target miR-635. miR-635 is situated on chromosome 17q and has a reduced expression in nonsmall cell lung cancer [6] and osteosarcoma tumor [7]; it can inhibit proliferation, migration of tumor cells, and other malignant phenotypes, thereby acting as a tumor suppressor gene in tumors. Until now, it is still unknown whether miR-635 has influence on the occurrence and development of myeloma. Since myeloma RPMI8226 cells have been extensively studied, their research characteristics have long been confirmed. Therefore, this study took myeloma RPMI8226 cells as the research object and mainly explored the effect of circ_0058063/miR-635 axis on malignant phenotype (proliferation, apoptosis, migration, and invasion) of myeloma cells and the possible mechanism, aiming to provide targeted molecular therapy of myeloma a new target.

## 2. Materials and Methods

### 2.1. Clinical Record

A collection of 47 patients with multiple myeloma who were diagnosed and treated in our hospital from December 2016 to October 2019, 25 males and 22 females, were involved, their average age is about 62.13 ± 9.12 years old. Inclusion criteria: initial diagnosis; no chemotherapy or radiotherapy before surgery. Exclusion criteria: patients with other malignant tumors; patients with chronic diseases such as hypertension and diabetes. Another 47 h matrix metalloproteinase 2 (MMP-2) healthy individuals who underwent bone marrow aspiration and had no abnormalities in bone marrow function at our institution during the same period were included as controls, who were 24 men and 23 women; their average age is about 59.46 ± 8.76 years old. The ethics committee of our hospital has approved this research, and the patients voluntarily signed the informed consent.

### 2.2. Cells and Reagents

Myeloma cell line RPMI8226, Guangzhou Jennio Biotech Co., Ltd.; fetal bovine serum (FBS), American HyClone Company; RPMI 1640 medium, Annexin V-FITC/PI Apoptosis Kit, and Bicaquinoline Acid (BCA) Protein Detection Kit, Beijing Solarbio Science and Technology Co., Ltd.; Lipofectamine™ 2000 kit, American Invitrogen Company; RNA drawer kit, reverse transcription kit, and PCR kit, Dalian Takara Company; PCR primers, circ_0058063 small interfering RNA (si-circ_0058063), out-of-order nonsense negative sequence (si-NC), miR-635 mimics (mimics), mock control sequence (miR-NC), circ_0058063 wild-type plasmid (WT-circ_0058063), mutant plasmid (MUT-circ_0058063), miR-635 inhibitor (anti-miR-635), and inhibitor negative sequence (anti-miR-NC), Sangon Biotech Shanghai Co., Ltd.; rabbit anti-human proliferating nuclear antigen Ki-67, B lymphocyte tumor-2 (Bcl-2), B lymphocyte tumor-2-related protein (Bax), MMP-9, and glyceraldehyde-phosphate dehydrogenase (GAPDH) polyclonal antibody, Santa Cruz Biotechnology, Inc.; dual luciferase activity detection kit, Promega Corporation.

### 2.3. Methods

#### 2.3.1. RT-qPCR Method to Test circ_0058063 and miR-635 Expression

Use RNA drawer reagent to extract total RNA from tissue, reverse transcription into cDNA, and perform PCR amplification. The amplification program is 95°C for 5 minutes, 95°C for 10 s, 60°C for 30 s, and 72°C for 30 s; the total cycles number must be 35. Primer sequence is as follows: circ_0058063 upstream 5′-TATGATCCTGTTTGGTGGTCGGCA-3′, downstream 5′-TGGACCAAGATGGGTAGCTTGTGA-3′; miR-635 upstream 5′-TATAGCATATGCAGGGTG-3′, downstream 5′-CGCATTCGGAGTGCGAGTT-3′; GAPDH upstream 5′-CTCGCTACACCTCAATACATCG-3′; downstream 5′-GCGCCATAAGTCTAGTATTGAGA-3′ U6 upstream 5′-GTACGACATACGACATAAC-3′, downstream 5′-CGACATACGAAGTGACGATG-3′. 2^−ΔΔCT^ method is to calculate the expression level of circ_0058063 relative to the internal control GAPDH and miR-635 relative to the internal control U6. ΔCt (*n*) = Ct target gene (*n*) − Ct internal reference gene (*n*); ΔΔCT (*n*) = ΔCt (*n*) − ΔCt (1).

#### 2.3.2. Cell Culture and Transfection

RPMI8226 cells were resuscitated and they were cultured with RPMI 1640 medium containing 10% FBS. RPMI8226 cells which are in the logarithmic growth phase were placed into a 6-well plate at 1.0 × 10^5^ cells/well and transfected with si-NC (si-NC group) and si-circ_0058063 (si-circ_0058063 group) using Lipofectamine^TM^ 2000 liposome, miR-NC (miR-NC group), miR-635 mimics (miR-635 group), cotransfection si-circ_0058063, and anti-miR-NC (si-circ_0058063 + anti-miR-NC group), si-circ_0058063, and anti-miR-635 (si-circ_0058063 + anti-miR-635 group). After 6 h of transfection, the medium was changed. After culturing for another 24 hours, RT-qPCR was used to detect circ_0058063 or miR-635 expression in each group of cells to verify the transfection effect. The method was the same as that in Section 2.3.1, and the cells were collected for subsequent experiments.

#### 2.3.3. CCK-8 Method to Test Cell Proliferation

Each cells group was placed into 96-well plates at 1.0 × 10^4^ cells/well and cultivated 24 hours. Each well adds 10 *μ*L of CCK-8 reagent. After 2 hours' incubating, the optical density (OD) value was measured with a microplate reader at 450 nm.

#### 2.3.4. Flow Cytometry to Test Apoptosis

Each cells group was placed in a 24-well plate at 5.0 × 10^4^ cells/well; after 24-hour cultivation, all the cells were collected. The cells were washed twice with PBS, 500 *μ*L binding buffer was added, and the cells were suspended. Annexin V-FITC/PI kit and flow cytometry were used to detect cell apoptosis.

#### 2.3.5. Transwell Method to Test Cell Migration and Invasion

The cell density of each group was adjusted into 5 × 10^4^ cells/mL. Migration experiment: the Transwell chamber was placed in one 24-well plate, 100 *μ*L cell suspension was added into the upper chamber and another 500 *μ*L culture medium was added into the lower chamber. After 24 hours' cultivation, the medium was discarded and fixed with 4% paraformaldehyde for half an hour, and at the same time 0.4% crystal violet was stained for 15 minutes. We observed under the microscope, randomly selected 5 samples of view, and counted the number of migrated cells. Invasion test: we spread the Transwell upper chamber with Matrigel ahead of time, kept it air-dried naturally and added 100 *μ*L of cell suspension, and then managed the subsequent operations according to the abovementioned migration experiment.

#### 2.3.6. Western Blot Method to Detect Ki-67, Bax, Bcl-2, MMP-2, and MMP-9 Protein Expression in Cells

We inoculated each group of cells in a 6-well plate at 1.0 × 10^5^ cells/well and collected the cells after culturing for 24 hours. RIPA reagent extracts total protein in cells, BCA method was to detect protein content, and then electrophoresis was performed by 12% SDS-PAGE. After electrophoresis, we wet transferred the protein isolate into PVDF membrane and adopted 5% skimmed milk powder solution to seal for 1 hour. The primary antibodies were added, Ki-67 (1 : 500), Bax (1 : 1000), Bcl-2 (1 : 1000), MMP-2 (1 : 500), MMP-9 (1 : 500), and GAPDH (1 : 1000), respectively. We incubated overnight at 4°C in the primary antibody incubation solution. Then, we put them in goat anti-rabbit secondary antibody (1 : 2000) incubation solution and incubated at 37°C for one hour. The developers were added to avoid light for development and we took photos with the gel system exposed.

#### 2.3.7. Dual Luciferase Reporter Gene Experiment

We seeded RPMI8226 cells into one 6-well plate at 1.0 × 10^5^ cells/well, and WT-circ_0058063 and miR-635 mimics or miR-NC, MUT-circ_0058063, and miR-635 mimics were cotransfected with Lipofectamine^TM^ 2000 liposome method. After 6 hours of transfection, we changed the medium. We incubated for another 24 h, collected and lysed the cells, under the operation of 3500 r/min, centrifuged for 5 min, and kept the supernatant. Refer to the instructions of the dual luciferase activity detection kit to detect the supernatant luciferase activity.

### 2.4. Statistical Analysis

We adopt SPSS 22.0 software to operate statistical analysis. Measurement data are expressed in the form of mean ± standard deviation ($\bar{x}$ ± *s*). To know about comparison between the abovementioned two groups, we use the independent sample *t*-test; as for multiple groups, we use the one-way analysis of variance and further pairwise comparisons and we use the SNK-q test. *P* < 0.05 means that the difference is statistically significant.

## 3. Result

### 3.1. circ_0058063 and miR-635 Expression in Multiple Myeloma

To make a comparison with normal bone marrow tissue, circ_0058063 expression in multiple myeloma tissue was increased (*P* < 0.05), but miR-635 expression in multiple myeloma tissue was decreased (*P* < 0.05). See Figure 1.

### 3.2. Knocking Down circ_0058063 Effect on Myeloma RPMI8226 Proliferation

circ_0058063 expression which transfected with si-circ_0058063 in RPMI8226 cells is significantly lower than being transfected with si-NC (*P* < 0.05), indicating that the construction of RPMI8226 cells that knocked down circ_0058063 was successful. Contrast with the si-NC group, the OD value and Ki-67 protein expression of RPMI8226 cells in the si-circ_0058063 group reduced (*P* < 0.05), indicating that knocking down circ_0058063 can inhibit the RPMI8226 cells proliferation. See Figure 2.

### 3.3. Knocking Down circ_0058063 Effect on the Apoptosis of Myeloma RPMI8226 Cells

Contrast with the si-NC group, RPMI8226 apoptotic rate together with Bax protein expression in the si-circ_0058063 group raised (*P* < 0.05), and Bcl-2 protein expression reduced (*P* < 0.05), indicating that knocking down circ_0058063 can promote RPMI8226 cells apoptosis. See Figure 3.

### 3.4. The Effect of Knockdown circ_0058063 on Myeloma RPMI8226 Cells Migration and Invasion

Contrast with the si-NC group, RPMI8226 cells migration and invasion quantities and MMP-2 together with MMP-9 proteins expression of the si-circ_0058063 group decreased (*P* < 0.05), indicating that knocking down circ_0058063 can inhibit the RPMI8226 cells migration and invasion. See Figure 4.

### 3.5. circ_0058063 Targeted Regulation of miR-635 Expression

Circular RNA Interactome bioinformatics software predicts that there are continuous binding sites between the nucleotide sequence of circ_0058063 and miR-635. Compared with WT-circ_0058063 cotransfected cells and miR-NC, the luciferase activity of cells cotransfected with WT-circ_0058063 and miR-635 mimics decreased (*P* < 0.05); compared with WT-circ_0058063 cotransfected cells and miR-NC, the luciferase activity of WT-circ_0058063 cotransfected cells and miR-635 mimics did not change significantly (*P* > 0.05), indicating that circ_0058063 can target miR-635, see Figure 5. At the same time, contrast with the si-NC group, miR-635 expression level of RPMI8226 cells in the si-circ_0058063 group was increased (2.91 ± 0.25 vs. 0.98 ± 0.06, *t* = 22.520, *P* < 0.05), further indicating that circ_0058063 targeted binding and negatively regulated miR-635 expression.

### 3.6. miR-635 Overexpression Effect on Myeloma RPMI8226 Proliferation, Apoptosis, Migration, and Invasion

miR-635 expression in RPMI8226 cells transfected with miR-635 mimics was significantly higher than that with miR-NC (*P* < 0.05), indicating that RPMI8226 cells overexpressing miR-635 were successfully constructed. Compared with the group pf miR-NC, the OD value, number of migration and invasion of RPMI8226 in the group of miR-635, and Ki-67, MMP-2 plus MMP-9 proteins expression reduced (*P* < 0.05), but the apoptosis rate and Bax protein expression raised (*P* < 0.05) and Bcl-2 protein expression reduced (*P* < 0.05), it means that miR-635 overexpression has the ability to inhibit proliferation, migration, and invasion of RPMI8226 cells and promote their apoptosis. See Figures 6 and 7.

### 3.7. Knockdown miR-635 Reverses Knockdown circ_0058063 Effect on Myeloma RPMI8226 Proliferation, Apoptosis, Migration, and Invasion

Compared with the group of si-circ_0058063 + anti-miR-NC, the expression level of miR-635 in RPMI 8226 cells in the si-circ_0058063 + anti-miR-635 group reduced (*P* < 0.05), and the cell OD value, the number of migration and invasion, and Ki-67, and MMP-2 plus MMP-9 protein expression raised (*P* < 0.05); in the meantime apoptosis rate and Bax protein expression reduced (*P* < 0.05), Bcl-2 protein expression raised (*P* < 0.05); it means knockdown miR-635 could reverse knockdown circ_0058063 inhibitory effect on RPMI8226 proliferation, migration, and invasion and the promotion of apoptosis. See Figures 8 and 9.

## 4. Discussion

circRNA has a closed circular and stable structure and is conservative. circRNA can play the role of miRNA molecular sponge, regulate miRNA target gene expression and then affect the process of cell proliferation, differentiation, and apoptosis, and affect the occurrence and development of multiple myeloma and other tumors [8]. Studies have shown that multiple circRNAs are not normally expressed in multiple myeloma tissues or patient plasma and are involved in regulating the development of multiple myeloma. For example, circ-CDYL is significantly increased in multiple myeloma cells and patient plasma, knockdown of circ-CDYL can significantly hinder the growth of multiple myeloma, and also the mechanism of action is linked with the targeted regulation of miR-1180/YAP axis. We can adopt circ-CDYL to become such potential therapeutic target for MM [9]. circ_0000190 is downregulated in both bone marrow tissue and peripheral blood of patients with multiple myeloma. circ_0000190 overexpression can target miR-767-5p and upregulate MAPK4 expression to inhibit the viability and proliferation and induce apoptosis of multiple myeloma. It could inhibit myeloma growth and development in the body [10]. circ-SMARCA5 expression decreased in multiple myeloma cell lines, and its overexpression can target and downregulate the expression of miR-767-5p, inhibit multiple myeloma proliferation, and promote apoptosis [11].

This study showed that circ_0058063 expression in multiple myeloma tissue was obviously higher than that in normal bone marrow tissue; knockdown of circ_0058063 effectively attenuates multiple myeloma proliferation, migration, and invasion and also promotes apoptosis, which is consistent with the obvious overexpression of circ_0058063 in bladder cancer tissue reported by Sun et al. [12]. Downregulation of circ_0058063 can target miR-145-5p/CDK6 axis to weaken bladder cancer proliferation and migration ability in vitro and also promote apoptosis. These results are consistent, suggesting that circ_0058063 promotes the development of multiple myeloma, which can be used as a treatment for these tumor potential molecular targets.

Ki-67 is involved in regulating the production cycle of tumor cells and is a marker protein of tumor cell proliferation [13]. MMP-2 plus MMP-9 are family members of MM. They take part in the degradation of extracellular matrix and basement membrane and promote tumor cell migration and invasion [14]. Bax/Bcl-2 is an apoptosis regulatory protein. When Bax expression increases, homodimers are formed, which changes the structure of cell mitochondrial membranes, resulting in cytochrome C's release, activates the caspase cascade, and induces apoptosis in turn, but when the expression of Bcl-2 increases, it forms a heterodimer with Bax, which weakens the proapoptotic effect of Bax and inhibits cell apoptosis [15]. This research shows that knocking down circ_0058063 can reduce the Ki-67, MMP-2, MMP-9, and Bcl-2 protein expression in multiple myeloma cells and promote the expression of Bax protein, suggesting that circ_0058063 may directly or indirectly regulate the expression of proteins related to proliferation, apoptosis, migration, and invasion and influence the malignant phenotype of multiple myeloma cells and thus affect the occurrence and development of multiple myeloma.

In order to further explore the molecular mechanism of knockdown circ_0058063 inhibiting the malignant phenotype of multiple myeloma cells, this research proved that circ_0058063 binds to the target and negatively regulates miR-635. The expression of miR-635 is reduced in a variety of tumors, exerting a tumor suppressor effect. Studies have shown that miR-635 is underexpressed in gastric cancer tissues and cell lines, and the low expression of miR-635 is closely related to the poor prognosis of patients with gastric cancer. Overexpression of miR-635 can target to inhibit the expression of KIFC1 and reduce the proliferation, migration, and invasion of gastric cancer cells [16]; The expression of miR-635 in osteosarcoma tissues was significantly reduced, the proliferation and invasion ability of osteosarcoma cells transfected with miR-635 mimics was weakened, and apoptosis increased, and transfection of miR-635 mimic can inhibit the growth of osteosarcoma in vivo [17]. miR-635 expression in multiple myeloma tissue is markedly lower than normal bone marrow tissue, and overexpression of miR-635 can inhibit the malignant phenotype of multiple myeloma cells, suggesting that miR-635 is also a tumor suppressor gene for multiple myeloma; the gene function may provide a new target for the treatment of multiple myeloma. Knockdown of miR-635 reversed the inhibitory effect of circ_0058063 on multiple myeloma proliferation, migration, and invasion and also the apoptosis promotion, further suggesting that circ_0058063 affects the progression of myeloma through targeted binding and negative regulation of the expression of miR-635.

In summary, the expression of circ_0058063 raised in multiple myeloma tissues, while miR-635 expression reduced. Knockdown of circ_0058063 can effectively reduce multiple myeloma proliferation, migration, and invasion and promote cell apoptosis. Its mechanism may be related to targeted binding and negative regulation of miR-635. The circ_0058063/miR-635 axis may provide a potential new target for the treatment of multiple myeloma. This study only explored the influence of the circ_0058063/miR-635 axis on the malignant phenotype of multiple myeloma cells through in vitro cell experiments. Next, we will further explore the miR-635 target genes and downstream signaling pathways about the occurrence and development of multiple myeloma. circ_0058063/miR-635 axis effect on multiple myeloma occurrence and development was verified in vivo by nude mouse transplantation tumor experiment.

## Figures and Tables

**Figure 1:** circ_0058063 and miR-635 expression in multiple myeloma ($\bar{x}$ ± *s*, *n* = 47). Contrast with normal bone marrow tissue, ^*∗*^*P* < 0.05.

**Figure 2:** Knockdown circ_0058063 effect on RPMI8226 cell proliferation ($\bar{x}$ ± *s*, *n* = 9). (a) circ_0058063 mRNA expression in multiple myeloma; (b) OD value; (c) Ki-67 protein expression in multiple myeloma. Contrast with si-NC group, ^*∗*^*P* < 0.05.

**Figure 3:** Knockdown circ_0058063 effect on RPMI8226 cell apoptosis ($\bar{x}$ ± *s*, *n* = 9). (a) Flow cytometric diagram of RPMI8226 cell apoptosis after circ_0058063 knockdown; (b) Bcl-2 and Bax protein expression in RPMI8226 cells after knocking down circ_0058063. Contrast with si-NC group, ^*∗*^*P* < 0.05.

**Figure 4:** Knockdown circ_0058063 effect on RPMI8226 migration and invasion ($\bar{x}$ ± *s*, *n* = 9). (a) RPMI8226 cell migration and invasion after knocking down circ_0058063; (b) MMP-2 together with MMP-9 protein expression for RPMI8226 after knocking down circ_0058063. Contrast with the group of si-NC, ^*∗*^*P* < 0.05.

**Figure 5:** circ_0058063 targeted regulation of miR-635 expression. Contrast with the group pf miR-NC, ^*∗*^*P* < 0.05.

**Figure 6:** miR-635 overexpression effect on RPMI8226 apoptosis, migration, and invasion ($\bar{x}$ ± *s*, *n* = 9). (a) miR-635 mRNA expression in multiple myeloma; (b) OD value; (c) flow cytometric diagram of RPMI8226 cell apoptosis after overexpression of miR-635; (d) RPMI8226 cell migration and invasion after miR-635 overexpression. Compared with the group of miR-NC, ^*∗*^*P* < 0.05.

**Figure 7:** RPMI8226 Ki-67, Bcl-2, Bax, MMP-2, and MMP-9 protein expression after miR-635 overexpression ($\bar{x}$ ± *s*, *n* = 9). Compared with the group of miR-NC, ^*∗*^*P* < 0.05.

**Figure 8:** Knockdown of miR-635 reverses the knockdown circ_0058063 effect on RPMI8226 apoptosis, migration, and invasion ($\bar{x}$ ± *s*, *n* = 9). (a) miR-635 mRNA expression in multiple myeloma; (b) OD value; (c) flow cytometric diagram of RPMI8226 cell apoptosis after miR-635 and circ_0058063 are knocked down at the same time; (d) after miR-635 and circ_0058063 were knocked down at the same time, RPMI8226 cells migrated and invaded. Contrast with si-circ_0058063 + anti-miR-NC group, ^*∗*^*P* < 0.05.

**Figure 9:** RPMI8226 Ki-67, Bcl-2, Bax, MMP-2, and MMP-9 protein expression after miR-635 and circ_0058063 are knocked down at the same time ($\bar{x}$ ± *s*, *n* = 9). Compared with the group of si-circ_0058063 + anti-miR-NC, ^*∗*^*P* < 0.05.

## Data Availability

The original data used to support the results of this study can be obtained from the corresponding author.
